# Serum thrombospondin-2 is a candidate diagnosis biomarker for early non-small-cell lung cancer

**DOI:** 10.1042/BSR20190476

**Published:** 2019-07-26

**Authors:** Yi-ming Jiang, Dan-lu Yu, Guo-xin Hou, Jia-lu Jiang, Qiang Zhou, Xiao-fang Xu

**Affiliations:** 1 Internal Medicine-Oncology, The First Hospital of Jiaxing, Jiaxing city, Zhejiang province 314001, China; 2 Endocrine Department, The First Hospital of Jiaxing, Jiaxing city, Zhejiang province 314001, China

**Keywords:** Biomarker, Diagnosis, NSCLC, Serum, THBS2

## Abstract

Thrombospondin-2 (THBS2) is a secreted protein overexpressed in numerous cancers and may function as a diagnostic tumor marker. The objective of the present study was to investigate the diagnostic performance of serum THBS2 in early stage non-small-cell lung cancer (NSCLC). Serum THBS2 and Cyfra21-1 level were evaluated in blood samples of 112 patients from NSCLC groups and 51 healthy control (HC) groups. Receiver operator characteristic (ROC) curves were used to evaluate the diagnostic significance. Serum THBS2 level was significantly up-regulated in NSCLC patients compared with healthy control subjects (*P*<0.0001), and the postoperative THBS2 level decreased significantly (*P*<0.0001). ROC curves analysis demonstrated that THBS2 was a comparable biomarker as Cyfra21-1 to distinguish early stage NSCLC or lung squamous cell carcinoma (SC) from healthy control subjects. And Cyfra21-1 was observed with significantly improved performances by the combination of THBS2 to distinguish early stage NSCLC (*P*<0.05) as well as SC (*P*<0.05) from the control subjects. In addition, THBS2 was estimated to perform well in the diagnosis of patients with Cyfra21-1-negative NSCLC (area under the curve [AUC] = 0.73). In summary, the present study suggested that serum THBS2 might be an early diagnostic biomarker for NSCLC.

## Introduction

Lung cancer is the leading causes of cancer death in the world. Non-small-cell lung cancer (NSCLC) accounts for about 80% of all cases of lung cancer and comprises primarily two histological types: adenocarcinoma (AC) and squamous cell carcinoma (SC) [1]. If diagnosed at the localized stage, the survival rates for NSCLC are much higher than that of with metastasis disease. Although new therapies have improved the outcomes of patients with NSCLC, the predicted 5-year survival rate is only about 16% [1]. Thus, detection of NSCLC at an early stage is of great significance for improving lung cancer prognosis. The utilization of imaging techniques, especially low-dose computed tomography (CT) scanning, has shown good potential for early diagnosis of NSCLC. However, the risk of radiation-induced lung cancer associated with repeated low-dose CT lung screening may not be negligible, especially for smokers or other high-risk populations [2]. Due to the lack of non-invasive and convenient tools, early diagnosis of NSCLC remains poor. Recently, it has been reported that noninvasive blood tests are widely accepted and become more and more appealing in NSCLC diagnosis.

Attempts have been made for the early detection of NSCLC by using blood biomarkers that indicate the presence of tumors [3,4]. Cyfra21-1, carcinoembryonic antigen (CEA), squamous cell carcinoma antigen (SCC) and tissue polypeptide antigen (TPA) are biomarkers being applied in the clinical diagnosis of NSCLC. However, the sensitivity and specificity are unsatisfactory, especially for the diagnosis of early stage NSCLC [5–7]. Therefore, it is crucial to explore novel biomarkers that can improve the diagnostic performances for early NSCLC with satisfactory sensitivity and specificity.

THBS-2 (also known as TSP-2) is a 150 kDa calcium-binding protein released from various types of cell, including stromal fibroblasts and endothelial cells. It is involved in multiple cellular activities including cytoskeletal organization, motility, angiogenesis and apoptosis [8–10]. Notably, the role of THBS2 in tumor cells has received more and more attention. In many tumors, the expression of THBS2 in tissues is associated with tumor progression and overall survival [11]. Moreover, THBS2 in peripheral blood also has a potential value of clinical application. Plasma THBS2, in combination with CA19.9, can help to detect early stage pancreatic ductal AC [12]. Microarray gene-expression and in-depth proteomic analysis have revealed that THBS2 is significantly up-regulated in NSCLC tissues [13–15]. However, the clinical significance of circulating THBS2 level in NSCLC has not yet been fully evaluated. In the present study, we detected serum THBS2 level in early stage NSCLC patients and assessed its potential as early diagnostic biomarkers for NSCLC.

## Materials and methods

### Patients and specimens

Blood samples from 51 healthy control subjects and 112 NSCLC patients prior to treatment were collected at The First Hospital of Jiaxing Hospital. The disease stages were determined according to the American Joint Committee on Cancer (AJCC) TNM (tumor–node–metastasis) classification [16], and limited to stage I and stage II. Age and sex matched volunteers without respiratory diseases were selected as healthy control subjects. Twenty postoperative blood samples were collected 2 weeks after tumor resection. Blood samples were centrifuged and the serum was aliquoted and snap frozen at −80°C until use. Clinical parameter data, including gender, age, histological subtype and clinical stage, were collected and summarized in Table 1. Informed consent was obtained from all individual participants of the present study. All procedures conducted in studies involving human participants are in accordance with the 1964 Helsinki Declaration and its subsequent revisions or similar ethical standards

**Table 1:** Characteristics of study participants

Diagnosis	Healthy control	Lung cancer
Sex		
Male	30	60
Female	21	52
Age		
Mean age	56	59
Range	22–65	24–72
Histological subtype		
AC	-	56
SC	-	56
Disease stage		
Stage I	-	21
Stage II	-	91

### Serum THBS2 detection by ELISA

THBS2 level in serum samples was measured by ELISA (R&D System Inc., MN, U.S.A.), according to the manufacturer’s instructions. In brief, a microtiter plate coated with capture antibody was incubated with 100 μl serum from NSCLC patients and healthy control subjects for 1 h at 37°C. After washing, the detection antibody was added and incubated for 30 min at room temperature. Adequate washing was carried out after each step. Following avidin-horseradish peroxidase-conjugated secondary antibody and TMB substrate solution, stop solution was added to terminate the reaction. The absorbance was determined at 450 nm using a Model 680 microplate reader (Bio-Rad, Hercules, CA). Analyze each sample in duplicate.

### Serum assays for Cyfra21-1

Serum Cyfra21-1 was measured by the Roche Cobas E601 immunoassay analyzer (Roche Diagnostics, Mannheim, Germany) according to the manufacturer’s instructions.

### Statistical analysis

SPSS 20.0 software (SPSS Inc., Chicago, IL, U.S.A.) and GraphPad software (GraphPad Software Inc., La Jolla, CA, U.S.A.) were used to analyze all data for statistical significance. All data are presented as mean ± SEM. Mann Whitney–Wilcoxon test was used for continuous variables. Paired Student’s *t-*test was performed to ascertain statistical significance between the preoperative and postoperative level of THBS2. Pearson’s correlation coefficient was used to evaluate the correlation of the two markers. Receiver operating characteristic (ROC) curves were plotted to assess diagnostic performance. The area under the curve (AUC) and 95% confidence interval were used to assess the discriminatory power. Comparison between related ROC curves was performed as described [17]. Values of *P*<0.05 were considered statistically significant.

## Results

### Increased serum level of THBS2 in patients with early stage NSCLC

First, Serum THBS2 level in early stage NSCLC patients and healthy control subjects were measured using ELISA kit. As shown in Figure 1A, the mean level of THBS2 in NSCLC patients was significantly higher than that in healthy control subjects (*P*<0.0001). Moreover, THBS2 was also observed with significantly higher level in two main histological types of NSCLC of AC (*P*<0.001) and squamous cell carcinoma (SC, *P*<0.0001) than that in healthy control subjects. However, there was no obvious difference between the two subtypes. The performance of THBS2 in the diagnosis of early stage NSCLC was assessed in a comparable manner. The level of cyfra21-1 which was a routinely clinical used biomarker for NSCLC was also evaluated. As reported, the level of cyfra21-1 in NSCLC patients is significantly up-regulated, and more pronounced in squamous cell carcinoma (Figure 1B). To determine how the serum biomarkers behaved in the diagnosis of early stage NSCLC, scatter plots of serum THBS2 and Cyfra21-1 levels were made and statistically analyzed (Figure 2). There was no correlation between serum THBS2 and Cyfra21-1 levels, with a correlation coefficient (r) of 0.18 (*P*=0.01). The results above indicated that serum THBS2 possesses potential ability to distinguish early stage NSCLC patients from healthy control subjects.

**Figure 1:** Increased serum level of THBS2 and Cyfra21-1 in early stage NSCLC patients (**A**) serum THBS2 level in healthy control subjects (*n*=51), patients with NSCLC (*n*=112), AC (*n*=56) and squamous cell carcinoma (SC, *n*=56). (**B**) serum Cyfra21-1 level in healthy control subjects (*n*=51), patients with NSCLC (*n*=112), AC (*n*=56) and squamous cell carcinoma (SC, *n*=56).

**Figure 2:** Correlation analysis of serum THBS2 and Cyfra21-1 No correlation between serum THBS2 and Cyfra21-1 (correlation coefficient, 0.18; *P*<0.01).

### Effect of surgical resection of NSCLC on serum THBS2 level

It has been reported that THBS2 is significantly up-regulated in NSCLC tissues [13,14]. To further verify that NSCLC tissue is the source of THBS2 in peripheral blood, we compared serum THBS2 level before and after surgery. Blood samples were collected 2 weeks after surgery from 20 NSCLC patients with relatively high level of THBS2. As shown in Figure 3, although the mean postoperative THBS2 level was much higher than the healthy control subjects (41.52 ± 9.87 vs 29.46 ± 9.00), it did decrease significantly (65.44 ± 7.44 vs 41.52 ± 9.87, *P*<0.0001).

**Figure 3:** Comparison of serum THBS2 level in patients with NSCLC pre- and postoperation The statistical difference was analyzed using the paired *t* test (*n*=20).

### Diagnostic performances of THBS2 and Cyfra21-1 for early stage NSCLC

Diagnostic performances of serum THBS2 and Cyfra21-1 for early stage NSCLC were evaluated by ROC curves analysis (Figure 4A and Table 2). The area under the curve (AUC), sensitivity, specificity, and all cut-off value of THBS2 and Cyfra21-1 levels were all determined using ROC analysis and summarized in Table 2. THBS2 predicted the present of NSCLC with an AUC of 0.74 (95% CI: 0.66–0.80) at a cut-off point of 31.88 ng/ml. This cut-off provided 72.32% sensitivity and 70.59% specificity. Meanwhile, Cyfra21-1 discriminated early NSCLC from healthy control subjects with an AUC of 0.82 (95% CI: 0.75–0.88) at a cut-off value of 2.69 ng/ml, which is lower than the clinical used value (3.30 ng/ml). As an individual marker, the performance of THBS2 was comparable with Cyfra21-1 in discriminating healthy control subjects versus early stage NSCLC (Figure 4A and Table 2). Moreover, the marker panel composed of THBS2 and Cyfra21-1 significantly improved the performance of Cyfra21-1 as individual biomarkers (AUCCyfra21-1 = 0.82 vs AUCTHBS2 + Cyfra21-1 = 0.87, *P*<0.05).

**Figure 4:** Diagnostic performances of THBS2 and Cyfra21-1 for early stage NSCLC Performances of THBS2 and Cyfra21-1 as individual markers and markers panel for discriminating NSCLC (**A**), AC, (**B**), squamous cell carcinoma (SC), (**C**) and Cyfra21-1-negative NSCLC patients (**D**) from healthy control subjects.

**Table 2:** Performances of THBS2 and Cyfra21-1 for NSCLC

	AUC (95% CI)	Sensitivity (%)	Specificity (%)	Cut-off value
HC vs NSCLC				
THBS2	0.74 (0.66–0.80)	72.32	70.59	31.88
Cyfra21-1	0.82 (0.75–0.88)	56.25	94.12	2.69
THBS2 + Cyfra21-1	0.87 (0.81–0.92)*	78.57	90.20	
HC vs AC				
THBS2	0.69 (0.59–0.78)	69.64	70.59	31.88
Cyfra21-1	0.77 (0.67–0.84)	83.93	60.78	1.55
THBS2 + Cyfra21-1	0.82 (0.73–0.88)	69.64	90.20	
HC vs SC				
THBS2	0.79 (0.70–0.86)	67.86	82.35	37.75
Cyfra21-1	0.88 (0.80–0.93)	69.64	94.12	2.69
THBS2 + Cyfra21-1	0.93 (0.86–0.97)*	85.71	90.20	
HC vs Cyfra21-1-negative NSCLC				
THBS2	0.73 (0.64–0.81)	73.44	70.59	31.88

* *P*<0.05 in comparison with Cyfra21-1.

As two main histological types of NSCLC, lung AC and squamous cell carcinoma (SC) exhibit different characteristics in the expression of tumor markers. Although with relatively unsatisfactory performance in discriminating AC from the control subjects (AUC = 0.69), THBS2 was observed with remarkable capability to distinguish SC from healthy control subjects, with an AUC of 0.79 (Figure 4B,C and Table 2). Notably, the distinguishing ability of Cyfra21-1 was also dramatically improved by the combination of THBS2 (AUCCyfra21-1 = 0.88 vs AUCTHBS2 + Cyfra21-1 = 0.93, *P*<0.05).

It should be noticed that if use the clinical used value of 3.30 ng/ml as the cut-off point of Cyfra21-1, as many as 64 NSCLC patients will be missed diagnosis. In order to make up for this deficiency of Cyfra21-1, we assessed the performance of THBS2 for those Cyfra21-1-negative NSCLC patients. As shown in Figure 4D, the AUC for THBS2 to distinguish Cyfra21-1-negative NSCLC patients from healthy control subjects are 0.73 (95% CI: 0.64–0.81).

## Discussion

THBS2 has been reported with debated and controversial roles in tumors occurrence and prognosis. On the one hand, it is reported that THBS2 plays protective roles in the tumorigenesis of many cancers and its expression is inversely correlated with vascularity of glioma [18], skin cancer [19], NSCLC [20], and colon cancer [21]. In addition, THBS2 has inhibitory effects on the metastasis of malignant melanoma [22] and pancreatic cancer [23]. However, it is also found that THBS2 was able to promote tumor metastasis by inducing matrix metalloproteinase-13 production in lung cancer cells [24]. Recently, THBS2 in peripheral blood has a potential value of clinical application attracted researcher attention. In pancreatic cancer, Kim et al. [12] found that the level of THBS2 in the plasma was significantly up-regulated, especially in the advanced stages of tumors, with good diagnosis performances for the malignant disease in combination with CA19.9. Fei et al. [25] reported that THBS2 as diagnosis serum biomarkers for CRC (colorectal cancer), which might be a good supplement for CEA or CA19-9 for clinical diagnosis. Wang et al. [26] also revealed that THBS2 might become as a potential biomarker for predicting clinical outcome for colorectal cancer patients. Diametrically opposite effects of down-regulation of THBS2 on the prognosis of patients have also been reported in gastric cancer [27,28] and colorectal cancer [29]. Those facts illustrate that the exact roles and clinical values of THBS2 in tumors remain to be further revealed.

Few studies have focused on the clinical significance of circulating THBS2. In the present study, the diagnostic performance of serum THBS2 for early stage NSCLC was evaluated, compared and combined with another biomarker, Cyfra21-1, which is already widely used in clinical practice. Receiver operator characteristic (ROC) curves analysis revealed that THBS2 was a comparable biomarker as Cyfra21-1 to distinguish early stage NSCLC or SC from healthy control subjects. Combined with THBS2, the performance of Cyfra21-1 was significantly improved. Moreover, THBS2 could also reduce the rate of missed diagnosis by the application of Cyfra21-1 alone.

Our data demonstrated that the postoperative level of THBS2 in NSCLC patients underwent tumor resection decreased significantly, which suggests that high level of THBS2 in peripheral blood are probably derived from the tumor tissue itself, as have been reported [13,14]. However, it should also be noticed that the mean postoperative THBS2 level was much higher than that of the healthy control subjects. Possible reasons are as follows: the postoperative blood samples were collected 2 weeks after surgery, and this time interval may be too short for the THBS2 protein in the blood to fully degraded, especially taken into consideration the fact that polymorphisms in thrombospondin genes could increase the conformational stability of the proteins [30]. It is necessary to detect the postoperative THBS2 level at extended time points, 2 months, for example, to determine whether it will return to normal level in future. And it is also essential to decide whether THBS2 can be used for disease recurrence monitoring.

Combined application of multiple markers is one of the important strategies for improving early diagnosis of lung cancer. Clinical used biomarker for lung cancer including CEA, squamous cell carcinoma antigen (SCC) and TPA, as well as Cyfra21-1. As is known that TPA and Cyfra21-1 are biomarkers with more diagnostic value for lung squamous cell carcinoma other than AC [31]. This could be attributed to the fact that TPA and Cyfra21-1, belonging to type II cytokeratin family, are generally released during cell death, which is more persistent and intense in squamous cell carcinoma [32]. Although there was no statistical difference between the mean level of THBS2 in AC and SC, it has been proved that diagnosis performance of THBS2 for SC is superior to AC, not only as an individual biomarker, but also in combination with Cyfra21-1. The performances of THBS2 combined with other markers of lung cancer require further study in the future.

In conclusion, our findings revealed that circulating THBS2 might serve as promising biomarkers for early detection of NSCLC.

## Abbreviations

AC: adenocarcinoma
AUC: area under the curve
CEA: carcinoembryonic antigen
CRC: colorectal cancer
CT: computed tomography
HC: healthy control
NSCLC: non-small-cell lung cancer
ROC: receiver operator characteristic
THBS2: thrombospondin-2
TPA: tissue polypeptide antigen
